# Tumor specific mutations in TERT promoter and CTNNB1 gene in hepatitis B and hepatitis C related hepatocellular carcinoma

**DOI:** 10.18632/oncotarget.9801

**Published:** 2016-06-02

**Authors:** Francesca Pezzuto, Francesco Izzo, Luigi Buonaguro, Clorinda Annunziata, Fabiana Tatangelo, Gerardo Botti, Franco M. Buonaguro, Maria Lina Tornesello

**Affiliations:** ^1^ Molecular Biology and Viral Oncology Unit, Istituto Nazionale Tumori “Fondazione G Pascale” - IRCCS, Napoli, Italy; ^2^ Hepatobiliary Surgery Unit, Istituto Nazionale Tumori “Fondazione G Pascale” - IRCCS, Napoli, Italy; ^3^ Department of Pathology, Istituto Nazionale Tumori “Fondazione G Pascale” – IRCCS Napoli, Italy

**Keywords:** hepatocellular carcinoma, TERT promoter, CTNNB1, hepatitis virus, Pathology Section

## Abstract

Recurrent somatic mutations in the promoter region of telomerase reverse transcriptase (TERT) gene and in the exon 3 of CTNNB1 gene have been recognized as common events in hepatocellular carcinoma (HCC) with variable frequencies depending on etiology and geographical region. We have analyzed TERT promoter and CTNNB1 gene mutations in 122 cases of hepatitis B (HBV) and hepatitis C (HCV) related HCCs, in 7 cases of cholangiocarcinoma (CC) and hepatocholangiocarcinoma (HCC-CC) as well as in autologous cirrhotic tissues. Overall, 50.4% and 26% of HCC as well as 14.3% and none of CC and HCC-CC were mutated in TERT promoter and in CTNNB1 exon 3, respectively. TERT and CTNNB1 mutations were found more frequently in HCV related (53.6% and 26.4%, respectively) than HBV related (41.7% and 16.7%, respectively) HCCs and coexisted in 57.6% of CTNNB1 mutated tumors. Mutations in TERT and CTNNB1 were not associated with the functional promoter polymorphism rs2853669. No mutations were detected in the 129 non-HCC cirrhotic tissues. In conclusion, mutations in TERT promoter and in CTNNB1 gene represent specific cancer signatures in the pathogenesis of viral related HCC and could be promising early biomarkers as well as targets for tailored therapies.

## INTRODUCTION

Primary liver cancer is the sixth most common tumor in the world with 782,000 new cases and 746,000 deaths in 2012, of which above 80% occur in less developed countries [1]. In Europe the highest incidence has been reported in Southern regions (age standardized rate [ASR] = 7.1 per 100,000 population in Italy) and the lowest in the Northern (ASR = 1.7 cases per 100,000 population in Iceland) [1]. An exceptional high incidence (ASR = 34.8 cases per 100′000 men) has been reported in Southern Italy [2].

Hepatocellular carcinoma (HCC), arising from hepatocytes, represents the dominant histotype of primary liver cancer accounting for 70%-85% of all cases worldwide [3]. Cholangiocarcinoma (CC), arising primarily from the biliary epithelium within the liver or the biliary tract, and hepatocholangiocarcinoma (HCC-CC), a combined liver and bile duct carcinoma, are relatively rare [4–6]. Hepatitis B (HBV) and hepatitis C (HCV) infections represent the major risk factors for HCC being associated with more than 80% of liver cancer cases worldwide [7]. The relative contribution of each virus varies in different geographic regions. Indeed, HBV is the major cause of HCC in Asia, Africa and Latin America and HCV the predominant cause of HCC in Europe and United States [8–10]. In Southern Italy 23.2% of men aged 65 years or older are HCV-positive [11] and over 60% of HCC cases develop on cirrhosis caused by chronic HCV infection [12].

HBV and HCV promote oncogenesis through a complex multistep process involving inflammation, hepatic damage, cirrhosis, increased liver fibrosis and HCC [13]. Viral, host and environmental co-factors contribute to the accumulation of multiple genetic alterations and growth advantage of transformed hepatocytes [14–15]. The TP53 oncosuppressor and CTNNB1 oncogene have been recognized as the most frequently mutated genes in HCC [16, 17]. More recently, high throughput sequencing allowed to uncover novel recurrent mutations in tumor driver genes and several deregulated pathways including Wnt/β-catenin, cell cycle, chromatin remodeling gene, histone methyltransferase, AKT/mTOR and RAS/RAF/MAP kinase [18–24].

Telomerase activation and telomere maintenance causing prolonged cell survival is a common feature of human tumors [25]. Several studies showed that short telomeres and reduced telomerase activity are markers of liver cirrhosis [26–28]. Instead, TERT activity is restored in up to 90% of HCC, compared to the 21% of non-tumor tissue [29–31]. The mechanisms of TERT reactivation have been only partially elucidated. Some studies showed that in HBV-related HCC there is a recurrent integration of viral genome nearby TERT gene and consequent telomerase reactivation in a significant number of cases [32, 33]. Recently, activating mutations have been identified by whole genome sequencing analysis at 124 bp (mostly G > A and rarely G > T) and 146 bp (G > A) before the ATG start site in the promoter region of TERT gene in several human tumors including melanoma, glioblastoma, bladder cancer, anaplastic thyroid cancer and HCC [34–37]. These mutations cause upregulation of TERT transcription by generating a binding site for ETS (E-twenty six) and ternary complex factor (TCF) transcription factors [38]. TERT promoter mutations have been also identified as a frequent genetic alteration in dysplastic hepatocellular nodules arising in cirrhosis and as a key event in malignant transformation of hepatocellular adenoma [23, 39, 40]. Several studies described variable distribution of TERT mutations in different geographical regions, reporting higher frequencies in HCC cases from Western countries (54-60%) and lower in Eastern countries (29-31%), and in HCC with different etiologies [22, 23, 41–43].

Recently the rs2853669 A > G single nucleotide polymorphism (SNP), located −245 bp upstream of the TERT gene ATG site, has shown to modulate TERT mRNA expression levels induced by TERT promoter somatic mutations [44]. Ko et al. showed that TERT mRNA levels were significantly higher in cell lines and HCC tumors harboring a combination of rs2853669 G allele and TERT promoter mutations compared to tumors with rs2853669 G allele only [45]. In addition, the rs2853669 G variant in combination with somatic variations was associated with increased mortality and higher cancer recurrence rate in HCC patients [45].

TERT promoter mutations have been found significantly associated with activating mutations in CTNNB1 gene, encoding for β-catenin, suggesting a cooperation between the two pathways [23]. Activation of the Wnt/β-catenin pathway plays an important role in hepatocarcinogenesis. Non-synonymous mutations at codons 31, 33, 37 and 45 of CTNNB1 exon 3 may cause loss of phosphorylation consensus sites at the N-terminus of β-catenin protein and consequent impairment of its degradation mediated by GSK3b/APC/axin complex [46]. CTNNB1 mutations have been identified more frequently in HCV-related than in HBV-related HCC [16, 17], and mainly associated with more advanced stages of malignant transformation [47].

In the present study, we evaluated genotype distribution of TERT rs2853669 polymorphism and the frequency of somatic mutations in TERT promoter and in exon 3 of CTNNB1 gene in a series of HCV- and HBV-positive cases diagnosed with HCC or CC/HCC-CC, along with autologous non-tumor tissue, from people living in Southern Italy, a geographic area with a very high incidence of liver cancer.

## RESULTS

### Somatic mutations and rs2853669 polymorphism in TERT promoter

Among 134 patients with liver cancer, 110 cases were HCV-related HCC, 12 HBV-related HCC and seven cases were CC/HCC-CC (Table 1). The mean age was 67.6 years (SD ±7.9) and the majority of patients were males (78%). Most of the patients had a single tumor (67.2%) and less than 5 cm in size (59.7%).

Overall 65 (48.5%) liver cancer cases were found positive for TERT promoter mutations comprising 64 out of 127 (50.4%) HCC and 1 out of 4 (25%) CC. HCV related HCC were significantly more frequently mutated (53.6%) than HBV-related (41.6%) HCCs, (*p* < 0.001). TERT promoter mutations were absent in the three HCC-CC and in 5 non-viral HCC tested in this study. Both hot spot mutations at nt −124 (G > A) and nt −146 (G > A) located upstream of the TERT ATG were identified in this cohort and found mutually exclusive. The nucleotide change at nt −124 was the most frequent representing 96.9% of all TERT mutations, while the mutation at nt −146 was found in only two cancer cases from male patients older than 65 years, of which one was positive for HCV and the second positive for HBV. All nucleotide mutations were heterozygous with only one affected allele (Figure 1). A total of 129 viral related cirrhosis autologous tissues along with 11 liver biopsies from non-tumor patients were analyzed for TERT promoter mutations and found all negatives. No sample showed the substitution A to C at nt −57, previously found in melanoma and in bladder cancer, or the tandem GG > AA mutations, described in melanoma.

**Table 1:** Characteristics of HCC, HCC-CC and CC patients

Characteristics	HCC (*n*=127) (%)	HCC-CC (*n*=3) (%)	CC (*n*=4) (%)	Normal Liver (*n*=11) (%)
**Sex**				
Males	97(76.4)	3(100)	2(50.0)	3(27.3)
Females	30(23.6)	0	2(50.0)	8(72.7)
**Age**				
<60	22(17.3)	0	0	2(18.2)
≥60	105(82.7)	3(100)	4(100)	9(81.8)
**Tumor size**				
<5 cm	68(53.5)	2(66.6)	2(50.0)	
≥5 cm	59(46.4)	1(33.3)	2(50.0)	
**Grading**				
G1	1(0.78)		0	
G2	122(96.1)	3(100)	4(100)	
G3	3(2.36)		0	
G4	1(0.78)		0	
**Staging**				
< Stage III	62(48.8)	1(33.3)	1(25.0)	
≥ Stage III	65(51.2)	2(66.6)	3(75.0)	
**AFP**				
≤20 ng/ml	52(40.9)	0	3(75.0)	
>20 ng/ml	75(59.0)	3(100)	1(25.0)	
**Tumor sites**				
Single	86(67.7)	2(66.6)	2(50.0)	
Multiple	41(32.3)	1(33.3)	2(50.0)	
**Etiology**				
HBV+	10(7.9)	1(33.3)	0	
HCV+	110(86.6)	2(66.6)	4(100)	
HBV+/HCV+	2(1.6)	0	0	
No viral	5(3.9)	0	0	

**Figure 1:** Representative sequence electropherograms of hot spot mutations at −124 and −146 bp and rs2853669 polymorphism at −245 bp from the ATG start site in TERT promoter

Similar frequencies of TERT mutations have been found in men (49%) and in women (46.8%), as well as in patients with single (48.8%) and multiple (47.7%) tumor sites. Higher mutation frequencies have been identified in HCV-related (53.6%) compared to HBV-related (41.7%) tumors, in patients with α-fetoprotein ≤20ng/ml (56.4%) *versus* those > 20ng/ml (43.1%), and in smaller tumors (52.7%) *versus* larger tumors (43.5%), however such differences did not reach statistical significance.

The TERT promoter SNP rs2853669 genotypes were analyzed in 84 HCC. The frequencies of −245 AA, −245 AG and −245 GG genotypes in HCC cases with mutated TERT promoter were 30.4% (*n* = 14), 45.6% (*n* = 21), 23.9% (*n* = 11) and among non mutated were 44.7% (*n* = 17), 39.5% (*n* = 15), 15.8% (*n* = 6), respectively. The rs2853669 genotype frequencies were in Hardy-Weinberg equilibrium in non mutated TERT cases (χ2 = 2.33; df = 1; *p* = 0.752) but were not in equilibrium among mutated TERT cases (χ2 = 6; df = 1; *p* = 0.014) suggesting a selective pressure of combined TERT promoter mutations and rs2853669 GG genotype in the latter group. The frequencies of rs2853669 GG and GA genotypes were more prevalent in TERT mutated HCC cases (69.6%) compared with controls (55.3%), although the difference did not reach statistical significance (*p* = 0.1789).

The survival analysis showed no correlation between the presence of TERT promoter mutations, alone or in combination with rs2853669 GG and GA genotypes, and poor prognosis.

### CTNNB1 mutations in liver cancer and association with TERT promoter mutations

Nucleotide changes affecting exon 3 of CTNNB1 gene were identified in 33 out of 134 (24.6%) liver cancer cases. Non-viral etiology and HCV-related HCC were more frequently mutated (40% and 26.4%, respectively) compared to HBV-related (16.7%) HCC. All identified mutations were heterozygous and located between codons 32 and 45. No insertions or deletions were identified. The majority of nucleotide changes occurred at codons 37 (39.4%), 33 (21.2%) and 45 (15.2%) and mainly affected serine residues. No CTNNB1 mutations were identified in CC/HCC-CC cases as well as in autologous control tissues and liver samples from healthy subjects. Among the 33 CTNNB1 mutated cases 19 (57.6 %) harbored also mutations in TERT promoter. Patients with both mutations were mostly men and all cases were HCV positive (Table 2).

Mantel-Cox log rank test showed that patients with CTNNB1 mutated cancers had a reduced survival compared to not-mutated, suggesting a correlation between CTNNB1 mutations and poor prognosis (*P* = 0.036; Mantel-Haenszel hazard ratio [HR] 3.73; 95% confidence intervals [CI] (Figure 2).

**Table 2:** Characteristics of patients according to the presence of TERT promoter (−124 G>A and −146 G>A) and CTNNB1 exon 3 mutations

Characteristics	TERT −124 G>A and −146 G>A	*P*	CTNNB1 exon 3	*P*
	(*n* = 65) (%)		(*n* = 33) (%)	
**Sex**		0.832		0.680
Males (*n* = 102)	50 (49.0)		26 (25.5)	
Females (*n* = 32)	15 (46.8)		7 (21.9)	
**Age**		0.437		0.754
≤ 60 (*n* = 22)	9 (40.9)		6 (27.3)	
> 60 (*n* = 112)	56 (50.0)		27 (24.1)	
**Tumor Size**		0.288		0.914
< 5 cm (*n* = 72)	38 (52.7)		18 (25.0)	
≥ 5 cm (*n* = 62)	27 (43.5)		15 (24.2)	
**Grading**		0.175		
G1 (*n* = 1)	1 (100)		1 (100)	0.246
G2 (*n* = 129)	63 (48.8)		31 (24.1)	0.596
G3 (*n* = 3)	0		1 (33.3)	1.000
G4 (*n* = 1)	1 (100)		0	1.000
**Staging**		0.173		0.267
<Stage III (*n* = 64)	35 (54.7)		13 (20.3)	
≥Stage III (*n* = 70)	30 (42.8)		20 (28.6)	
**AFP**		0.130		0.188
≤20 ng/ml (*n* = 55)	31 (56.4)		16 (29.1)	
>20 ng/ml (*n* = 79)	34 (43.1)		17 (21.5)	
**Tumor sites**		0.900		0.102
Single (*n* = 90)	44 (48.8)		26 (28.8)	
Multiple (*n* = 44)	21 (47.7)		7 (15.9)	
**Etiology**				
HCC HBV+ (*n* = 12)*	5 (41.7)	0.620	2 (16.7)	0.730
HCC HCV+ (*n* = 110)	59 (53.6)	<0.0001	29 (26.4)	0.320
HCC No viral (*n* = 5)	0	0.058	2 (40.0)	0.596
HCC-CC HBV+ (*n* = 1)	0		0	
HCC-CC HCV+ (*n* = 2)	0		0	
CC HCV+ (*n* = 4)	1 (25.0)		0	
**Event**		0.368		0.036^†^
Survival >2 years (*n* = 21)	13 (61.9)		9 (42.9)	

* This group comprises two cases of HBV+/HCV+ cases

† Log Rank test has been used to compare the survival distributions of mutated and non-mutated cases.

**Figure 2:** Survival percentages were compared using the Log-Rank Test (Mantel-Cox) **A.** HCC patients with TERT promoter mutations to those without mutations (median 36.4 *vs* 36.2 months, respectively; *P* = 0.368). **B.** HCC patients with and without TERT promoter mutations (median 36 *vs* 48 months, respectively; *P* = 0.036).

## DISCUSSION

Telomerase activity has been found up regulated in many human cancers denoting its crucial role in tumor development [37]. Somatic mutations and rs2853669 polymorphism in the promoter region of TERT gene have provided a genetic cause for telomerase activity [23, 39].

In this study we confirmed a high frequency of TERT promoter mutation in HCV-related HCC (53.6%). The overall mutation frequency detected in HCC from our series (50.4%) is lower than the one found in the French HCC series (59%) [42], but similar to the mutation frequency observed in Japan (54%) and USA (47%) [23, 37] and higher than the frequency reported in Taiwan (29%) and in Germany (44%) [41, 48].

In agreement with previous studies the G > A transitions at −124 bp (97%) before the TERT ATG start site was the most frequent nucleotide change. No mutations were identified in any matched peri-tumor cirrhotic tissue confirming the somatic nature of TERT promoter mutations and their very-likely driver function in neoplastic transformation.

The common polymorphism rs2853669 has shown to cause the inhibition of E2F1 transcriptional repressor and increased levels of TERT expression [45]. The combination of rs2853669 polymorphism and somatic TERT promoter mutations has reported to further increase TERT transcription levels and to be associated with higher risk of death and cancer recurrence in liver cancer patients [45]. The stratification of the data in our study did not show a significant effect of rs2853669 polymorphism and TERT promoter mutation on survival in HCC patients, however, rs2853669 alleles were not in Hardy Weinberg equilibrium among TERT mutated cases suggesting a selective pressure of rs2853669 allele G in tumors with both mutations.

TERT promoter mutations have been rarely found in liver cancer displaying biliary phenotype [48]. Fujimoto et al. analyzed the genetic landscape of 97 liver cancer of biliary origin and identified TERT mutations in 53% of CC/HCC-CC and only in 5.2% of CC [49]. We found no mutations in HCC-CC cases and only one TERT mutated case in CC confirming their cell type specificity in liver neoplastic tissue.

Aberrant activation of Wnt signaling and nuclear accumulation of β-catenin has been frequently reported in HCC [50]. Mutations in CTNNB1 mostly affect a β-catenin region rich in serine and threonine phosphorylation sites causing impaired Axin/APC/GSK3 mediated degradation and gain of oncogenic activity [46]. CTNNB1 mutations have been identified in about 20 - 40% of liver cancers [17, 51–53]. In our study, 29.7% of HCC were mutated in CTNNB1 between codon 32 and codon 45 and serine residues were the mostly affected amino acids (73% of mutations).

A recent meta-analysis including 2,334 liver cancer cases from 22 studies showed that accumulation of β-catenin in the cytoplasm and/or nucleus significantly correlated with vascular invasion and poor prognosis [54]. In our study CTNNB1 mutated cases had a reduced survival compared to not-mutated cases, supporting a correlation between mutations and outcome of disease (*P* = 0.036; Mantel-Haenszel HR 3.73; 95% CI 1.09 to 12.8). Additionally, CTNNB1 mutations have been found as an early alteration in a subset of hepatocellular adenomas transformed to HCC, while TERT promoter mutations were associated with late stages of adenoma to carcinoma transition suggesting an interplay between telomerase maintenance and Wnt/β-catenin pathway in last step of malignant transformation [42, 55]. The association between occurrence of mutations in CTNNB1 and TERT promoter has also been found in HCC [40]. We found that 57.6% of CTNNB1 mutated HCC also harbored activating mutations in TERT promoter.

One limitation of this study is that complete clinical information during the follow up was only available for a fraction of the patients, therefore a firm conclusion on the predictivity of TERT promoter and CTNNB1 mutations on the patient prognosis cannot be drawn. Nonetheless, our findings are consistent with other studies.

In conclusion, we present evidence that TERT promoter and CTNNB1 mutations have a high frequency in HCC of viral origin, particularly in HCV-related HCC, and are very specific to the tumor tissues given their constant absence in the autologous non-tumor cirrhotic tissues. Considering the high specificity and the earliness of TERT promoter mutations in liver cancer, we hypothesize their use as reliable biomarkers of HCC development in cirrhotic patients.

## MATERIALS AND METHODS

### Patients and tissue samples

A cohort of 145 consecutive patients surgically treated at the Hepatobiliary Unit of the National Cancer Institute “Fondazione Pascale” in Naples were enrolled in this study. Tumor biopsies from 110 HCV-positive HCC, 12 HBV-related HCC, four cases of CC and three cases of HCC-CC along with 134 autologous non-tumor tissue biopsies have been analyzed. Eleven biopsies from healthy patients have been also included in the analyses as control. Patients were classified according to Child -Pugh score into A (*n* = 114) and B (*n* = 23). Tumor size and number of tumor nodules were determined by computed tomography or magnetic resonance imaging. Each liver biopsy was divided in two sections: the first section was stored in RNA Later (Ambion, Austin, TX) at −80°C, the second was subjected to histopathologic examination. Similarly, autologous non-tumor biopsies were obtained from each patient, divided in two sections and processed for molecular analysis and histopathologic examination. Only liver biopsies histological confirmed to be hepatocellular carcinoma, cholangiocarcinoma, hepatocholangiocarcinoma or cirrhosis were included in the study. HCC were classified in four groups according to the histological grade: well differentiated (G1 *n* = 1), moderately differentiated (G2 *n* = 129) and poorly differentiated (G3 *n* = 3; G4 *n* = 1) according to the criteria of Edmondson and Steiner [56].

Tissue samples were digested with 150 μg/ml of proteinase K at 37°C for 12 hours in 100-500 μl of lysis buffer (10 mM Tris-HCL, pH 7.6, 5 mM EDTA, 150 mM NaCl, 1% SDS) followed by DNA purification with phenol-chloroform-isoamyl alcohol (25:24:1) extraction and ethanol precipitation in 0.3 M sodium acetate (pH 4.6). This study was approved by the Institutional Scientific Board and by the Ethical Committee of the Istituto Nazionale Tumori “Fond Pascale”, and is in accordance with the principles of the Declaration of Helsinki. All patients provided written informed consent.

### TERT promoter mutational analysis

TERT promoter region was amplified using the oligoprimers hTERT-F (5′-ACGAACGTGGCCAGCGGCAG-3′) and hTERT-R (5′-CTGGCGTCCCTGCACCCTGG-3′), which generate a 474 bp fragment covering the rs2853669 A > G SNP and hot spots −124 and −146 bp before TERT ATG. PCR negative samples were further amplified with oligonucleotides hTERT_short_F (5′- CAGCGCTGCCTGAAACTC-3′) and hTERT_short_R (5′- GTCCTGCCCCTTCACCTT-3′) targeting a shorter fragment of 163 bp covering the hot spots −124 and −146 bp in TERT promoter. PCR reactions were performed in 50 μL reaction mixture containing 300 ng of genomic DNA, 10 pmol of each primer, 1.25 Unit of Hot Master Taq DNA Polymerase (5 Prime GmbH, Hamburg, Germany) and 25 μl of PreMix J (Master Amp PCR, Epicentre). DNA was amplified in Sure Cycler 8800 thermal cycler (Agilent Technologies) with the following steps: an initial denaturation at 94°C for 3 minutes, followed by 45 amplification cycles of annealing at 65°C for 30 s, elongation at 72°C for 1 min, denaturation at 94°C for 30 s, and 10 min final elongation at 72°C. All samples were subjected to automated bidirectional direct sequencing analysis (Eurofins, Milan).

### CTNNB1 exon 3 mutational analysis

CTNNB1 exon 3 was amplified using the oligoprimers Beta-F (5′-CCAATCTACTAATGCTAATACTG-3′) and Beta-R (5′-GCATTCTGACTTTCAGTAAGCC-3′) able to generate a 310 bp fragment, which covers hot spot codons 33, 37, 41 and 45. PCR reactions and nucleotide sequencing were performed as previously described [17].

### Statistical analyses

Statistical analyses were performed using EpiInfo Versions 6 and Graphpad Prism 6 software. Patients were stratified by mutational status, sex, age, tumor grade and hepatitis virus infection. Comparison between groups was performed using Mantel Haenszel corrected χ^2^ test or Fisher exact test, as appropriate. Survival rates were estimated using the Log-Rank Test (Mantel-Cox). Overall survival was defined as the period between the time of surgery and death. Living patients were censored with the date of their last follow-up. *P*-values of less than 0.05 were considered statistically significant.

## Abbreviations

TERT: Telomerase reverse transcriptase
CTNNB1: β-catenin 1
HCC: hepatocellular carcinoma
CC: colangiocarcinoma
HCC-CC: hepato-cholangiocarcinoma
HBV: hepatitis B virus
HCV: hepatitis C virus
SNP: Single nucleotide polymorphism
